RETRACTED

# Prediction of Dissolved Oxygen Concentration in Sewage Treatment Process Based on Data Recognition Algorithm

**DOI:** 10.1155/2022/1525902

**Published:** 2022-06-24

**Authors:** Lili Ma, Jiangping Liu

**Affiliations:** College of Computer and Information Engineering of the Inner Mongolia Agricultural University, Hohhot 010018, China

## Abstract

In order to realize the real-time and accurate prediction of dissolved oxygen concentration in the sewage treatment process, a prediction model of dissolved oxygen concentration in the sewage treatment process based on a data identification algorithm was proposed. Combined with the data characteristics of the sewage treatment process, a new sample similarity measure is defined to extract more representative modeling data. In the improved algorithm, in order to improve the quality of the initial members of the basic fireworks algorithm, the chaos algorithm is integrated. The search mechanism of the basic fireworks algorithm is improved, and the optimization process is divided into two stages based on the set criteria, and two groups are used simultaneously. The results show that compared with the basic FWA algorithm, the CFWA algorithm makes better use of the chaotic search mechanism. On the one hand, it avoids the excessive random or blind selection of the initial weight threshold of the neural network in the initial stage; on the other hand, in the optimization process of the weight threshold, two types of search mechanisms, FWA and COA, are used to give full play to their respective strengths and to continuously conduct information exchange and mutual cooperation between groups and individuals. The number of times is better than the basic FWA algorithm, and the training error and generalization error of the CFWA model in the simulation results of the soft sensor model are also better than those of the FWA model, which fully verifies the effectiveness of the CFWA algorithm. It is proved that the data recognition algorithm can effectively predict sewage treatment. It is proved that the data recognition algorithm can effectively predict the dissolved oxygen concentration in wastewater treatment process. It provides a new measurement method for some key process variables that cannot be measured or are difficult to measure in complex chemical processes.

## 1. Introduction

Urban sewage treatment and recycling is one of the effective ways to improve the ecological environment and solve the problem of urban water shortage. At present, the biochemical method is mostly used in sewage treatment, which is the main way of industrial and urban sewage treatment. The monitoring and control of DO is very important to improve the treatment quality and efficiency of the sewage treatment process. The actual sewage treatment process has the characteristics of complex and changeable sewage components and large uncertainty of sewage sludge flow. The research on online soft sensing technology of DO and other parameters is of great significance [1]. This research is divided into two parts: the first part establishes the mathematical model of dissolved oxygen concentration in the sewage treatment system under ideal conditions. Then, according to the analysis of the controlled object, the data recognition algorithm is applied in the sewage treatment process, and the data recognition is used as the controller. The training error and generalization error of CFWA model are also better than those of the FWA model. The FWA model fully verifies the effectiveness of the CFWA algorithm and proves that the data identification algorithm can effectively predict the dissolved oxygen concentration in the sewage treatment process. It is used to reduce the cost of sewage treatment and improve the quality of the effluent.

RETRACTED

## 2. Literature Review

Farhi and others have successfully realized the control of aeration volume in the sewage treatment process by using fuzzy multilevel control. They mainly use fuzzy logic control to control the aeration time in the aeration tank so that the oxygen in the air can be fully utilized in the biochemical reaction process. The biggest advantage of the neural network is that it can fully approximate any nonlinear model and has been widely used in sewage treatment. For example, using the relationship between water quality parameters, the target value of each parameter can be predicted through the neural network, and the model of the system can also be identified [2]. Qaderi and others proposed a hybrid model for the anaerobic digestion process. The model is established based on the material balance equation, in which the biological growth rate is expressed by a neural network [3]. Zhang and others studied the dynamic simulation of the activated sludge process, used a neural network to improve the prediction model, and developed a program to improve the accuracy of the existing mechanical model of activated sludge process [4]. Wang and others studied the demand index of oxygen content in the process of water treatment and used the neural network to predict the grey model [5]. Manabu made an in-depth analysis of the complexity, uncertainty, and difficulty in establishing an accurate mathematical model of the urban sewage biological treatment system [6]. Gu et al. proposed a fuzzy controller using a neural network to complete rule reasoning. This control method enhances the accuracy of the control process to a certain extent [7]. Weng et al. believe that with the development of modern industry and the continuous growth of the urban population, more and more sewage discharge has not only caused great damage to the whole ecological environment but also caused a serious waste of resources, thus affecting people's normal life and work. In addition, due to the limited freshwater resources in China, many places require that the discharge of sewage treatment system must meet the reuse standard to realize the recycling of sewage treatment [8]. Li et al. believe that in order to ensure the sustainable development of China's economy, we must explore more advanced sewage treatment processes, technologies, and countermeasures to achieve effective treatment and recycling of sewage. At present, countries all over the world have increased the intensity and policies of sewage treatment and have more strict requirements for the discharge of industrial wastewater and domestic sewage, that is to say, they have higher standards for the effluent quality and treatment accuracy of sewage treatment [9]. Dou et al. believe that the impact load of the whole sewage treatment process leads to poor stability in the sewage treatment process because the inlet water quality and sewage flow of the sewage treatment plant change greatly with time, and the outlet water quality often does not meet the discharge standard, accompanied by sludge bulking. Therefore, if traditional methods are still used to control large-scale sewage treatment links, it is obvious that it cannot meet the needs of modern society [10].

RETRACTED

On the basis of the current research, this paper proposes a prediction model of dissolved oxygen concentration in the sewage treatment process based on a data identification algorithm. Combined with the data characteristics of the sewage treatment process, a new sample similarity measure is defined to extract more representative modeling data. In the improved algorithm, in order to improve the quality of the initial members of the basic fireworks algorithm, a new method is defined. The improved two-level sinusoidal chaotic map uses the ergodicity of chaotic motion to select the initial group members of the fireworks algorithm; the search mechanism of the basic fireworks algorithm is improved by fusing the chaotic algorithm, and the optimization process is divided into two stages based on the set criteria and adopts The two groups are carried out at the same time. The results fully verify the effectiveness of the CFWA algorithm. It is proved that the data identification algorithm can effectively predict the dissolved oxygen concentration in the sewage treatment process.

RETRACTED

## 3. Research Methods

### 3.1. Data Recognition Algorithm

The realization idea of the fireworks algorithm under the data recognition algorithm is to regard fireworks as a feasible solution in the solution space of the optimization problem. The process of a fireworks explosion producing a certain number of sparks is the process of neighborhood search for the optimal solution. The algorithm is described as follows:

(1) Randomly generate *N* fireworks, that is, randomly initialize *n* positions *x*_*i*_ in the solution space to represent *n* initial solutions of the problem.
(2) Calculate the fitness value of each firework, evaluate the quality of fireworks, and produce different quantities of sparks under different explosion radii. The calculation formulas of explosion radius *R*_*i*_ and explosion spark number *S*_*i*_ of fireworks *x*_*i*_ are as follows:
  (1) $$\begin{array}{c} R_{i}=R\times \frac{f\left(x_{i}\right)-y_{\min}+\varepsilon }{\sum_{i=1}^{N}\left(f\left(x_{i}\right)-y_{\min}\right)+\varepsilon }, \end{array}$$
  (2) $$\begin{array}{c} S_{i}=M\times \frac{y_{\max}-f\left(x_{i}\right)+\varepsilon }{\sum_{i=1}^{N}\left(y_{\max}-f\left(x_{i}\right)\right)+\varepsilon }, \end{array}$$
where *y*_min_=min(*f*(*x*_*i*_))(*i*=1,2,…, *N*) is the minimum fitness (optimal value) in the current fireworks population and *y*_max_=max(*f*(*x*_*i*_))(*i*=1,2,…, *N*) is the maximum fitness (the worst value) in the current fireworks population. The constants *R* and *M* are used to adjust the explosion radius and the number of explosion sparks, respectively, and *ε* is the small amount used to avoid division by zero. In addition, in order to limit the number of spark particles generated at the fireworks position with good fitness value and poor fitness value, the number of sparks is limited as follows:
  (3) $$\begin{array}{c} S_{i}=\left\{\begin{array}{cc} \text{round}\left(a\cdot M\right), & S_{i}<aM,\\ \text{round}\left(b\cdot M\right), & S_{i}<aM,\;a<b<1\\ \text{round}\left(S_{i}\right), & \text{other}. \end{array}\right., \end{array}$$
Here, *a* and *b* are two constants and round is the rounding function
(3) Generate explosive sparks and randomly select *z* dimensions to form a set DS, *z* = round (*D* × rand (0, 1)), where *D* represents the *x* dimension of fireworks, round is the function of rounding, and rand is the function of generating random numbers subject to a uniform distribution in the interval. Refer to equation (4) to conduct explosion operation on each dimension *k* of DS and save *ex*_*ik*_ in the explosion spark population after cross-border treatment.
  (4) $$\begin{array}{c} ex_{ik}=x_{ik}+h,\\ h=R_{i}\times \text{rand}\left(-1,1\right), \end{array}$$
where *h* represents position offset, *x*_*ik*_ represents the *k*-th dimension of the *i*-th fireworks individual, and *ex*_*ik*_ represents the explosion spark of *x*_*ik*_ after explosion operation [11].
(4) Generate *G* Gaussian variation sparks, randomly select spark *x*_*i*_, and randomly select *z* dimensions to form a set DS so that *z* = round (*D* × rand (0, 1)), where *D* represents the dimension of fireworks member *x*_*i*_. Referring to equation (5), perform Gaussian mutation operation on each dimension *k* of DS and save *mx*_*ik*_ in Gaussian mutation population after cross-border processing.
  (5) $$\begin{array}{c} mx_{ik}=x_{ik}\times e, \end{array}$$
where *e*∼*N* (1, 1) and *mx*_*ik*_ is the Gaussian variation spark generated after *x*_*ik*_ Gaussian variation.
(5) *N* members are selected from the three population members of fireworks, explosion sparks, and Gaussian variation sparks to form the fireworks population for the next iteration. Let the candidate set be *S* (including three types of population members), and the individual with the best fitness value in the fireworks population size of NS is first determined as the next generation of fireworks members, and the other *N*–1 fireworks members are selected from *s* in turn by roulette. The probability of candidate *x*_*i*_ being selected is
  (6) $$\begin{array}{c} p\left(x_{i}\right)=\frac{R\left(x_{i}\right)}{\sum_{x_{j}\in K}R\left(x_{i}\right)},\\ R\left(x_{i}\right)=\sum_{x_{j}\in K}d\left(x_{i}-x_{j}\right)=\sum_{x_{j}\in K}\left\|x_{i}-x_{j}\right\|, \end{array}$$
where *R*(*x*_*i*_) is the sum of the distance between each body in *x*_*i*_ and *S*. The higher the density of individuals in *S*, the lower the probability of being selected.
(6) Determine whether the termination conditions are met. If satisfied, stop the search; otherwise, return to step (2).

RETRACTED

### 3.2. Selection of Initial Fireworks Members

Therefore, the larger the size of fireworks members is, the more favorable it is, but it will also increase the computational complexity of the algorithm. According to the complexity of solving the problem, the group size is usually set to 10∼100. Conventional FWA selects the initial fireworks members randomly, which has certain blindness. When the solution space is large, it is difficult to ensure that a limited number of fireworks members are evenly distributed in the whole solution space, which increases the probability of the FWA algorithm falling into local optimization and is not conducive to improving the overall optimization efficiency of the algorithm. Chaos refers to a certain but unpredictable motion state. The motion ergodic characteristic can make chaotic variables traverse all states without repetition within a certain range according to their own “law” [12]. As shown in equation (7), a logistic map is a classical model for studying chaotic motion, which is in a completely chaotic state when *µ* = 4.

(7) $$\begin{array}{c} z_{n+1}=\mu z_{n}\left(1-z_{n}\right). \end{array}$$

The analysis and research show that the orbital points of chaotic variables generated by equation (7) are not evenly distributed, and there are problems of fixed points (multiple iterations approach a fixed value) and stability window (points gather in a certain interval). Based on the existing methods, this paper uses two-stage sinusoidal chaotic mapping to redistribute the fractal coefficients and defines an improved sinusoidal chaotic mapping SM:

(8) $$\begin{array}{c} z_{n+2}=r\;\sin\left(\frac{5.65}{z_{n+1}}\right)+\left(1-r\right)\sin\left(\frac{5.65}{z_{n}}\right),\;-1\leq z_{n}\leq 1,\;z_{n}\neq 0, \end{array}$$

where fractal coefficient *r*∼(0,1). When *r* = 0 or *r* = 1, the mapping is transformed into sinusoidal chaotic full mapping. In addition, the initial value *z*_0_ of the iteration cannot be 0, and *z*_0_ cannot be taken as any point of infinite equilibrium points; otherwise, chaos cannot be generated. The simulation shows that when *r* = 0.005, its randomness is basically close to the full map, and its chaotic characteristics are good, so *r* = 0.005 is taken in this paper. In order to improve the quality of FWA initial fireworks, the SM chaotic map defined in equation (8) is used to generate a large-scale initial population in the solution space, and the evenly distributed FWA initial fireworks are extracted from it according to the Euclidean distance between members so that the limited scale fireworks members are evenly distributed in the solution space [13]. The selection process of FWA initial fireworks members is described as follows:

1. Several different initial values are selected, and SM mapping is used for chaotic iteration. Depending on the size of the solution space, a multidimensional initial chaotic vector of a certain scale is generated, *X* ∈ *R*^*n*^, and *n* represents the dimension of the solution space;
2. Calculate the spatial distance (Euclidean distance) *d*_*ij*_ between vectors *X*_*i*_ and *X*_*j*_. If *d*_*ij*_ is less than the set threshold, eliminate one vector in *X*_*i*_ and *X*_*j*_ [14].

### 3.3. Performance Test

Simulation experiments are carried out to verify the effectiveness of the proposed hybrid algorithm. During the experiment, three optimization algorithms, particle swarm optimization (PSO), GA (genetic algorithm) and FWA, are introduced to compare with the improved chaotic fireworks hybrid optimization algorithm (CFWA). The optimization test objects are four classical functions (Ackley, Rastrigin, Griewank, and Rosenbrock) with multiple peaks, multiple local extremum points, and independent or interactive variables [15]. The global minimum value of *f*_1_(*x*) ~ *f*_3_(*x*) function is 0, and the corresponding optimal solution is *x*^*∗*^(0,0,…, 0). When the global minimum value of *f*_4_(*x*) function is also 0 and the corresponding optimal solution is *x*^*∗*^=(1,1,…, 1), the conventional PSO, GA, and FWA algorithms can quickly find the ideal solution for the four classical functions in the case of low dimension (such as 2∼3 dimensions) because there are few local extreme points. However, with the increase of dimension (such as more than 10 dimensions), the number of local extreme points increases sharply, and the optimization of the three basic optimization algorithms is more difficult [16].

RETRACTED

During the simulation analysis, the optimization accuracy settings of the four functions are 10^−6^, 10^−2^, 10^−2^, and 10^−2^. The population size of PSO, GA, FWA, and CFWA is 40, and the maximum number of iterations is set to 2,000. The other parameter settings are as follows:

FWA and CFWA: explosion radius adjustment constant *R* = 240, adjustment constant of explosion spark number *M* = 200, upper limit of explosive sparks am = 20, lower limit of explosive sparks bm = 1, and Gaussian variation spark number *G* = 50. The chaotic algorithm adopts the improved sinusoidal chaotic map SM proposed in this paper. See equation (8) for details. PPSO: c1 = c2 = 2.0, *ω*_max_=0.60, and *ω*_min_=0.06. GA: crossover probability is 0.6. The probability of variation is 0.01.

For the four optimization problems, the basic PSO, basic GA, basic FWA, and CFWA methods are used to randomly conduct 300 independent optimization tests.

## 4. Experiment and Analysis

A large sewage treatment plant is a complex engineering system with nonlinear, uncertain, large pure lag, strong coupling, distributed parameters, and hybrid system characteristics. As shown in Figure 1, the process of a sewage biochemical treatment enterprise is a typical predenitrification biological denitrification process [17]. Because it involves many subprocesses (reactions) such as physics, chemistry, and biology, the mechanism of the whole sewage biochemical treatment process is complex and diverse, and the material flow is interactive and coupled. In addition, with the change in seasonal temperature, the biological reaction rate is also different. DO is an important monitoring parameter in the process of sewage treatment, which is directly related to the effluent quality and control quality. Real time and accurate measurement of DO is the premise to improve the efficiency of sewage treatment and ensure the effluent quality. The analysis shows that there are many factors affecting DO, and the parameter value is subject to the superposition of various factors at any time. The research on online soft sensing technology of DO in the sewage treatment process is of great significance. Based on the process mechanism and empirical knowledge of the actual sewage biochemical treatment system, various factors affecting DO are deeply investigated and analyzed. The research shows that six parameters such as biochemical oxygen demand (BOD) and solid suspended solids have significant effects on DO value [18]. During soft sensing modeling, six auxiliary variables such as biochemical oxygen demand (BOD), suspended solids, total nitrogen mass concentration, total phosphorus mass concentration, chemical oxygen demand (COD), and influent flow are selected as the input variables of the model, and DO is the output variable of the model. In order to simplify the soft sensing model, the representative sample acquisition method proposed above is used for similarity analysis to remove the redundant samples in the sample set. The specific sample extraction method is described as follows:

After the sample normalization processing, the Euclidean distance, cosine distance, and corresponding *δ* value between two samples are calculated to obtain the *I* x *I* dimensional upper triangular square matrix *D*^*∗*^=(*δ*_*ij*_)_*l*×*l*_,  *l*=400,  *i*, *j*=1,…, *l*. When *i* > *j*,  *δ*_*ij*_=0, the threshold is set according to the actual situation of the preprocessed data, that is, when |*δ*_*ij*_| < 0.49, one sample is eliminated. After processing, the soft sensing modeling samples were reduced from 400 groups to 237 groups [19].

RETRACTED

An online soft sensing model of the sewage treatment process based on an artificial neural network (structure: 6-13-1; the total number of network weight thresholds is 105) is constructed. The offline training algorithm is the CFWA hybrid optimization algorithm proposed in this paper, and three optimization algorithms of basic PSO, GA, and FWA are introduced to compare with the improved algorithm. In the process of soft sensor modeling, the group member size of the four optimization algorithms is 50; the maximum number of iterations is 6,000; and the group member dimension is 105. Other experimental parameters are set as follows: FWA and CFWA, explosion radius adjustment constant *R* = 240, adjustment constant of explosion spark number *M* = 250, upper limit of explosive sparks am = 25, lower limit of explosive sparks BM = 1, and Gaussian variation spark number *G* = 60. The chaotic algorithm adopts the improved sinusoidal chaotic map SM proposed in this paper. PSO, c1 = c2 = 2.0, *ω*_max_=0.60,  *ω*_min_=0.06. GA: crossover probability is 0.6. The probability of variation is 0.01 [20].

In addition, for the selection of the initial weight threshold in neural network training, the existing methods mostly set the value range [−1∼+1]. The research shows that the selection of initial value has a certain impact on preventing local convergence and improving the convergence speed. Among them, the initial group members of basic PSO, GA, and FWA optimization algorithms are selected randomly. In the CFWA hybrid optimization algorithm, in order to ensure the quality of initial fireworks members, the defined SM chaotic map is used to generate an initial candidate group with a scale of 5,000 within the value range of weight threshold [−1∼+1], and then the initial fireworks members with uniform distribution and group scale of 50 are extracted according to the Euclidean distance between members [21]. At the end of the training, the optimal weight threshold is saved for online measurement of DO by the soft sensing model. Figures 2–5 show the analysis and comparison of the training and test results of the soft sensing model based on four algorithms. ER1 represents the root-mean-square error, and ER2 represents the average generalization error. The training and generalization effects of the soft sensor model based on the CFWA algorithm are shown in Figures 6 and 7, respectively.

The comparison results show that the soft sensing model based on the CFWA algorithm has lower training error and generalization error than the three basic soft sensing models of PSO, GA, and FWA. Its generalization ability is obviously better than the other three soft sensing models, and the accuracy is also greatly improved, which is consistent with the results of the performance test [22].

Compared with the basic FWA algorithm, the CFWA algorithm makes better use of the chaotic search mechanism. On the one hand, it avoids the excessive random or blind selection of the initial weight threshold of the neural network in the initial stage. On the other hand, in the optimization process of weight threshold, two types of search mechanisms, FWA and COA, are adopted to give full play to their respective strengths and continuously carry out information exchange and mutual cooperation between groups and individuals [23–26].

## 5. Conclusion

In this paper, an improved chaotic fireworks hybrid optimization algorithm is proposed, and a soft sensing model of dissolved oxygen mass concentration based on the improved algorithm is established. Aiming at the shortcomings of the existing FWA, an improved two-stage sinusoidal chaotic map is designed, and the initial member extraction method of FWA is improved by using the ergodicity of chaotic motion. In addition, in order to further improve the optimization performance of the existing FWA, the FWA algorithm and chaotic algorithm are organically integrated, making full use of their respective advantages, and based on the setting criteria, a chaotic fireworks hybrid optimization algorithm is proposed. Taking four classical high-dimensional complex functions as optimization objects, the optimization test of the improved algorithm is carried out. It provides a new measurement method for some key process variables that cannot be measured or are difficult to be measured in complex chemical processes.

RETRACTED

To sum up, through the analysis and research of the activated sludge wastewater treatment system, the paper proposes a control method, which achieves the expected control requirements, improves the treatment quality of the wastewater treatment system, and avoids oxygen in the control process. The waste of resources makes the whole sewage treatment process more economical. Due to the limited time and equipment, the research of the paper is not deep enough and needs to be further studied, mainly including the following parts:

1. More in-depth research is needed on the mathematical model of the sewage treatment system, and more accurate models are established in various sewage treatment links, so as to provide a reliable premise for the application of intelligent control methods.
2. In the case that the precise mathematical model of the sewage treatment system is unknown, the robustness of the control scheme during the training and learning process needs further research so that it can achieve higher control accuracy.

## Figures and Tables

**Figure 1:** Sewage treatment process flow.

**Figure 2:** PSO model simulation results.

**Figure 3:** GA model simulation results.

**Figure 4:** FWA3 model simulation results.

**Figure 5:** CFWA model simulation results.

**Figure 6:** Training results of dissolved oxygen mass concentration soft sensing model.

**Figure 7:** Generalization results of dissolved oxygen mass concentration soft sensing model.

## Data Availability

The data used to support the findings of this study are available from the corresponding author upon request.
